# Statistical Inference under Censored Data for the New Exponential-X Fréchet Distribution: Simulation and Application to Leukemia Data

**DOI:** 10.1155/2021/2167670

**Published:** 2021-08-29

**Authors:** Omar Alzeley, Ehab M. Almetwally, Ahmed M. Gemeay, Huda M. Alshanbari, E. H. Hafez, M. H. Abu-Moussa

**Affiliations:** ^1^Department of Mathematics, Umm Al-Qura University, Al-Qunfudah University College, Mecca, Saudi Arabia; ^2^Department of Statistics, Faculty of Business Administration, Delta University of Science and Technology, Mansoura, Egypt; ^3^Department of Mathematics, Faculty of Science, Tanta University, Tanta 31527, Egypt; ^4^Department of Mathematical Sciences, College of Science, Princess Nourah bint Abdulrahman University, Riyadh, Saudi Arabia; ^5^Department of Mathematics, Faculty of Science, Helwan University, Helwan, Egypt; ^6^Department of Mathematics, Faculty of Science, Cairo University, Giza, Egypt

## Abstract

In reliability studies, the best fitting of lifetime models leads to accurate estimates and predictions, especially when these models have nonmonotone hazard functions. For this purpose, the new Exponential-X Fréchet (NEXF) distribution that belongs to the new exponential-X (NEX) family of distributions is proposed to be a superior fitting model for some reliability models with nonmonotone hazard functions and beat the competitive distribution such as the exponential distribution and Frechet distribution with two and three parameters. So, we concentrated our effort to introduce a new novel model. Throughout this research, we have studied the properties of its statistical measures of the NEXF distribution. The process of parameter estimation has been studied under a complete sample and Type-I censoring scheme. The numerical simulation is detailed to asses the proposed techniques of estimation. Finally, a Type-I censoring real-life application on leukaemia patient's survival with a new treatment has been studied to illustrate the estimation methods, which are well fitted by the NEXF distribution among all its competitors. We used for the fitting test the novel modified Kolmogorov–Smirnov (KS) algorithm for fitting Type-I censored data.

## 1. Introduction

Modeling real-life events and natural processes using probability distributions is one of the most important processes in statistics and probability, where these processes are characterised by complexity and risk. For these reasons, statisticians have worked on the development of probability distributions, as proven probability distributions continue to fall short of accurately describing data obtained from natural events. These help to expand and modify probability distributions in generalized ways. Generalized probability distributions have emerged as a consequence of the widespread availability of additional parameters. Adding a special parameter to existing probability functions increases the precision of adequacy of the data obtained from natural phenomena as well as the accuracy of the distribution tail form's description.

In recent years, various research works were undertaken to create new distributions through creating new families and classes by modifying the baseline distribution by adding additional shape parameter(s). There are a large number of well-known classes of distribution that exist in the literature. For examples, see references [1–10].

One of the most well-known lifetime distributions is the exponential distribution, which has accordingly received considerable attention from statisticians. A superior novel family of distribution dubbed as a new exponential-X (NEX) family was introduced by Huo et al. [11]. It can model data with different shapes to their hazard function, such as increasing, decreasing, and bathtub. The distribution function (CDF) and density function (PDF) for the NEX family are defined as

(1) $$\begin{array}{c} G\left(x;\Theta \right)=1-\frac{1-F\left(x;\Omega \right)}{e^{\beta F\left(x;\Omega \right)}},\;x>0,\beta >0, \end{array}$$

(2) $$\begin{array}{c} g\left(x;\Theta \right)=f\left(x;\Omega \right)\frac{1+\beta \left[1-F\left(x;\Omega \right)\right]}{e^{\beta F\left(x;\Omega \right)}},\;x>0,\beta >0, \end{array}$$

where the vector of the parameters is denoted by Θ of the family. It consists of (Ω, *β*), which are the vectors of parameters for the baseline distribution and the additional shape parameter for the family, respectively.

The standard Fréchet distribution is a well-defined limiting distribution. It is commonly used to characterise variables associated with extreme phenomena like floods, rains, and cash flow. It was first introduced by Fréchet [12]. We can say that *X* is a random variable that has the two-parameter Fréchet distribution if its CDF and PDF are written as follows:

(3) $$\begin{array}{c} F\left(x;\Omega \right)=e^{-{\left(\alpha /x\right)}^{\lambda }},\;x>0,\beta >0,\\ f\left(x;\Omega \right)=\frac{\lambda }{x}{\left(\frac{\alpha }{x}\right)}^{\lambda }e^{-{\left(\alpha /x\right)}^{\lambda }},\;x>0,\alpha ,\lambda >0, \end{array}$$

where the vector of the parameters Ω=(*α*, *λ*) consists of the shape and scale parameters, respectively, for the Fréchet distribution.

The Fréchet distribution has received attention of a large number of authors such as Nadarajah and Kotz [13], where the standard Fréchet distribution is generalised as an exponentiated Fréchet distribution. Cordeiro et al. [14] discussed a new class of exponentiated generalised distributions, with regard to which functions such as the Exponentiated Generalised Fréchet, Exponentiated Generalised Normal, Exponentiated Generalised Gamma, and Exponentiated Generalised Gumbel have been introduced. A new lifetime distribution called the Weibull Fréchet distribution, which has four parameters, has been defined and studied by Afify et al. [15]. Teamah et al. [16] presented the Fréchet–Weibull distribution with application to earthquake datasets. Teamah et al. [17] introduced the Fréchet–Weibull Mixture Distribution. Almetwally and Muhammed [18] introduced a new novel bivariate distribution depending on copulas. Furthermore, Teamah et al. [19] presented a right truncated model of the Fréchet–Weibull Distribution. Mead et al. [20] introduced the beta exponential Fréchet distribution. The properties of the Gompertz Fréchet distribution have been studied by Oguntunde et al. [21]. An overview of the various estimators and applications for the Fréchet distribution has been discussed by Ramos et al. [22].

The innovations and encouragements to write this article are to introduce a new exponential-X Fréchet distribution as a good fit for the lifetime models that have increasing, decreasing, and bathtub failure rates. We have studied its mathematical properties such as its linear representation, quantile function, moments, generating function, incomplete moments, mean residual life and mean inactivity time, inequality curves, and order statistics. Furthermore, approaches to parameter estimation such as maximum likelihood, maximum product spacing, and Bayesian methods have been discussed using Type-I censored data. The Markov Chain Monte Carlo (MCMC) algorithm has been used as an approximation to Bayesian estimates. An extensive simulation study has been done. A comparison of the suggested estimate techniques has been conducted. Finally, the NEXF distribution has demonstrated its efficiency at fitting real-life data to a greater extent than other competitor distributions with regard to real-life applications.

The following is the structure of the paper: in Section 2, the proposed distribution is presented, and its behaviour is studied using different graphs. Various mathematical properties have been studied in Section 3.  Section 4 discusses the estimating techniques used to determine parameters.  Section 5 contains the interval estimation for the distribution's parameters. The simulation experiments have been performed, and its results were tabulated in Section 6. We worked on a real numerical example for the remission times as a data application, and this application is analyzed and fitted using the suitable fitting algorithm according to Type-I censoring in Section 7. After this, Section 8 contains the current study conclusions and other remarks.

### 1.1. Type-I Censoring Scheme

Assume that *n* identical components are arranged in a life testing experiment. We perform the experiment using a scheme of a Type-I censored sample. The test comes to an end at predetermined point in time *T*, and only the failure times prior to this time are recorded. Then, the number of units that fail by time *T*, say *m*, is a random variable, where *m* < *n*. The lifetimes of the initial *m* failures are determined, as well as the lifetimes of the subsequent *m* failures of the remaining *n* − *m* units are censored, where all that is known is that they will be greater than *T*. In this case, the model can be known as a Type-I censoring model (see Balakrishnan and Aggarwala [23]). For more examples of censored sampling based on different schemes, see [24–33].

Assume that the Type-I censored sample arises from CDF *F*(*t*) with PDF *f*(*t*). The joint density function of Type-I censored data, *x*_1:*n*_, *x*_2:*n*_,…, *x*_*m*:*n*_, is then given by

(4) $$\begin{array}{c} f\left(x_{1},x_{2},\ldots ,x_{m}\right)=\frac{n!}{\left(n-m\right)!}{\left[1-F\left(T\right)\right]}^{n-m}\prod_{i=1}^{m}f\left(x_{i}\right), \end{array}$$

where *x*_1_ < *x*_2_ < ⋯<*x*_*m*_ < *T* < *x*_*m*+1_.

## 2. The NEXF Distribution

Based on the NEX family with the Fréchet baseline distribution, we have obtained the NEXF distribution according to three parameters. We can derive easily the CDF and PDF of the NEXF distribution by the aid of the the Fréchet distribution and both equations (1) and (2), which can be given as follows:

(5) $$\begin{array}{c} G\left(x;\Theta \right)=1-\frac{1-e^{-{\left(\alpha /x\right)}^{\lambda }}}{e^{\beta e^{-{\left(\alpha /x\right)}^{\lambda }}}},\;x>0,\alpha ,\lambda ,\beta >0, \end{array}$$

(6) $$\begin{array}{c} g\left(x;\Theta \right)=\frac{\lambda }{x}{\left(\frac{\alpha }{x}\right)}^{\lambda }e^{-{\left(\alpha /x\right)}^{\lambda }}\frac{1+\beta \left[1-e^{-{\left(\alpha /x\right)}^{\lambda }}\right]}{e^{\beta e^{-{\left(\alpha /x\right)}^{\lambda }}}},\;x>0,\alpha ,\lambda ,\beta >0. \end{array}$$

We can say that a random variable *X* is distributed according to the NEXF distribution with PDF as in equation (6) by *X*∼NEXF(*α*, *β*, *λ*). The two-parameter NEX inverse Rayleigh model is a special case of the NEXF model obtained by letting *λ*⟶2.

The NEXF distribution's hazard rate function (HR) is provided by the following:

(7) $$\begin{array}{c} h\left(x;\Theta \right)=\frac{\lambda }{x}{\left(\frac{\alpha }{x}\right)}^{\lambda }e^{-{\left(\alpha /x\right)}^{\lambda }}\frac{1+\beta \left[1-e^{-{\left(\alpha /x\right)}^{\lambda }}\right]}{1-e^{-{\left(\alpha /x\right)}^{\lambda }}}. \end{array}$$

While its revised hazard rate function (RHR) can be written and defined by the following equation:

(8) $$\begin{array}{c} rh\left(x;\Theta \right)=\frac{\left(\lambda /x\right){\left(\alpha /x\right)}^{\lambda }e^{-{\left(\alpha /x\right)}^{\lambda }}\left(1+\beta \left[1-e^{-{\left(\alpha /x\right)}^{\lambda }}\right]\right)}{e^{\beta e^{-{\left(\alpha /x\right)}^{\lambda }}}+e^{-{\left(\alpha /x\right)}^{\lambda }}-1}. \end{array}$$

In order to make a reasonable study on the distribution, we chose different values for its parameters, and the graphs of its PDF and HR function are plotted in Figures 1 and 2 . From these figures, it may be noticed that the behaviour of the NEXF PDF curve may have different shapes. It may be skewed to right or even to left, or posses symmetric shape or declining shape, while the NEXF HR curves may be constant, decreasing, or upside down, which means that the proposed model is an attractive lifetime model. The NEXF distribution shows great flexibility in terms of its ability to model skewed data, as noted in the application section, so it sees widespread use in various fields such as biology, biomedical experiments, reliability, and survival studies.

## 3. Mathematical Properties

### 3.1. Linear Representation

The CDF of equation (1) is represented in the following form:

(9) $$\begin{array}{c} G\left(x\right)=1-\left[1-F\left(x\right)\right]e^{-\beta F\left(x\right)}=1-\overset{\infty }{\underset{k=0}{\sum }}\frac{{\left(-1\right)}^{k}\beta^{k}}{k!}\left[1-F\left(x\right)\right]F^{k}\left(x\right)\\ =1-\overset{\infty }{\underset{k=0}{\sum }}\overset{1}{\underset{m=0}{\sum }}\left(\begin{array}{c} 1\\ m \end{array}\right)\frac{{\left(-1\right)}^{m+k}\beta^{k}}{k!}F^{m+k}\left(x\right). \end{array}$$

By applying the previous expansion to the Fréchet distribution, we gain the CDF of the NEXF distribution in an expanded form as per the following:

(10) $$\begin{array}{c} F\left(x\right)=1-\overset{\infty }{\underset{k=0}{\sum }}\overset{1}{\underset{m=0}{\sum }}\left(\begin{array}{c} 1\\ m \end{array}\right)\frac{{\left(-1\right)}^{m+k}\beta^{k}}{k!}e^{-\left(m+k\right){\left(\alpha /x\right)}^{\lambda }}. \end{array}$$

By calculating the derivative of the above equation in terms of *x*, we can determine and easily find the PDF of the NEXF distribution in an expanded form as per the following:

(11) $$\begin{array}{c} f\left(x\right)=\overset{1}{\underset{m=0}{\sum }}\overset{\infty }{\underset{k=0}{\sum }}\left(\begin{array}{c} 1\\ m \end{array}\right)\frac{{\left(-1\right)}^{m+k+1}\beta^{k}}{k!}\frac{\lambda \left(k+m\right){\left(\alpha /x\right)}^{\lambda }e^{-\left(k+m\right){\left(\alpha /x\right)}^{\lambda }}}{x}=\overset{1}{\underset{m=0}{\sum }}\overset{\infty }{\underset{k=0}{\sum }}\Phi_{m,k}h_{m+k}\left(x\right). \end{array}$$

We can say that $\Phi_{m,k}=\left(\begin{array}{c} 1\\ m \end{array}\right)\left({\left(-1\right)}^{k+1}\beta^{k}/k!\right)$ and *h*_*m*+*k*_(*x*) is the Fréchet density function having a *α*[*m*+*k*]^1/*λ*^ as a scale parameter and a shape parameter *λ*.

### 3.2. Quantile Function QF

We can express and define the QF of the NEXF distribution as the inverse of the CDF of equation (5), and it is as follows:

(12) $$\begin{array}{c} Q\left(p\right)=\alpha {\left(\log\left\{\frac{\beta }{\beta -W\left[-e^{\beta }\beta \left(p-1\right)\right]}\right\}\right)}^{-\left(1/\lambda \right)},\;0<p<1, \end{array}$$

where *W*[·] is the Lambert function.

The NEXF distribution's 3 quartiles are determined by specifying special values for *p*, so when we set in equation (12) *p*=0.25 and 0.5, we get the first and second quartile, respectively, while when we set and *p*=0.75, we get the third quartile in equation (12).

Let *p*_*i*_ is distributed uniformly from 0 to 1, then the QF of the NEXF distribution can be adopted to generate a randomized sample that can be used in simulation and other applications throughout the following equation:

(13) $$\begin{array}{c} x_{i}=\alpha {\left(\log\left\{\frac{\beta }{\beta -W\left[-e^{\beta }\beta \left(p_{i}-1\right)\right]}\right\}\right)}^{-\left(1/\lambda \right)},\;i=1,2,\ldots ,n. \end{array}$$

### 3.3. The Moments

The most important thing for any distribution is to find its moments in an easy and simple ways. So, we can find the *r*th moments of the proposed NEXF distribution as shown in the following steps:

(14) $$\begin{array}{c} \mu_{r}^{\prime }=E\left(X^{r}\right)=\int_{0}^{\infty }x^{r}f\left(x\right)\text{d}x=\overset{1}{\underset{m=0}{\sum }}\overset{\infty }{\underset{k=0}{\sum }}\Phi_{m,k}\int_{0}^{\infty }x^{r}h_{m+k}\left(x\right)\\ =\overset{1}{\underset{m=0}{\sum }}\overset{\infty }{\underset{k=0}{\sum }}\Phi_{m,k}\Gamma \left(1-\frac{r}{\lambda }\right){\left[\alpha {\left[m+k\right]}^{1/\lambda }\right]}^{r},\;r<\lambda . \end{array}$$

By assigning *r*=1,2,3, and 4 in the preceding equation, we can drive the moments around the origin, from the first moment to the fourth moment, respectively.

We can derive the *n*^th^ central moment of the random variable *X*, say *μ*_*n*_, which is obtained as

(15) $$\begin{array}{c} \mu_{n}=E{\left(x-\mu \right)}^{n}=\overset{\infty }{\underset{k=0}{\sum }}{\left(-1\right)}^{k}\left(\begin{array}{c} n\\ k \end{array}\right)\mu_{1}^{\prime k}\mu_{n-k}^{\prime }. \end{array}$$

The cumulants (*k*_*n*_) of *X* can be found as follows:

(16) $$\begin{array}{c} k_{n}=\mu_{n}^{\prime }-\overset{n-1}{\underset{k=0}{\sum }}\left(\begin{array}{c} n-1\\ k-1 \end{array}\right)k_{r}\mu_{n-r}^{\prime }. \end{array}$$

### 3.4. Moment Generating Function (MGF)

We can write the MGF of the Fréchet distribution using the following equation:

(17) $$\begin{array}{c} M\left(t\right)=\int_{0}^{\infty }e^{tx}f\left(x\right)\text{d}x=\lambda \alpha^{\lambda }\int_{0}^{\infty }e^{tx}x^{-\lambda -1}e^{-{\left(\alpha /x\right)}^{\lambda }}\text{d}x, \end{array}$$

where by setting *y*=*x*^−1^ and by expanding the first exponential, we have

(18) $$\begin{array}{c} M\left(t\right)=\overset{\infty }{\underset{m=0}{\sum }}\frac{\alpha^{m}t^{m}}{m!}\Gamma \left(\frac{\lambda -m}{\lambda }\right). \end{array}$$

Assume that the right generalised hypergeometric function is described as follows:

(19) Ωqpα1,A1,…,αp,Apλ1,B1,…,λq,Bq;x=∑n=0∞∏j=1pΓαj+Ajnxn∏j=1qΓλj+Bjnn!.

As a result, we may write the MGF as

(20) Mt=Ω011,−λ−1−;αt.

Then, the MGF of the NEXF distribution can be written and defined as follows:

(21) Mt=∑m=01∑k=0∞Φm,kΩ011,−λ−1−;αm+k1/λt.

We may get and determine the formula for the proposed distribution's characteristic function simply by substituting *t* for it in the preceding equation.

### 3.5. The Incomplete Moments

One of the fundamental formulas is the incomplete moments, so this subsection is devoted to derive the formula of the *s*^th^ incomplete moment of the NEXF distribution:

(22) $$\begin{array}{c} \Psi_{s}\left(t\right)=\int_{0}^{t}x^{s}f\left(x\right)\text{d}x=\overset{1}{\underset{m=0}{\sum }}\overset{\infty }{\underset{k=0}{\sum }}\Phi_{m,k}\int_{0}^{t}x^{s}h_{m+k}\left(x\right)\\ =\overset{1}{\underset{m=0}{\sum }}\overset{\infty }{\underset{k=0}{\sum }}\Phi_{m,k}{\left(m+k\right)}^{s/\lambda }\gamma \left[1-\frac{s}{\lambda },\left(m+k\right){\left(\frac{\alpha }{t}\right)}^{\lambda }\right], \end{array}$$

such that *γ*(*a*, *z*) is the lower incomplete gamma function.

### 3.6. Mean Residual Life (MRL) and Mean Inactivity Time (MIT)

The MRL of the NEXF distribution is defined as follows:

(23) $$\begin{array}{c} \text{MRL}=\frac{1-\Psi_{1}\left(t\right)}{S\left(t\right)-t}=\frac{1-\sum_{m=0}^{1}\sum_{k=0}^{\infty }\Phi_{m,k}{\left(m+k\right)}^{s/\lambda }\gamma \left[1-\left(1/\lambda \right),\left(m+k\right){\left(\alpha /t\right)}^{\lambda }\right]}{\left[1-e^{-{\left(\alpha /x\right)}^{\lambda }}\right]e^{-\beta e^{-{\left(\alpha /x\right)}^{\lambda }}}-t}, \end{array}$$

where Ψ_1_(*t*) is the first incomplete moment of the NEXF distribution.

The MIT of the NEXF distribution is defined as follows:

(24) $$\begin{array}{c} \text{MIT}=t-\frac{\Psi_{1}\left(t\right)}{F\left(t\right)}=t-\frac{\sum_{m=0}^{1}\sum_{k=0}^{\infty }\Phi_{m,k}{\left(m+k\right)}^{s/\lambda }\gamma \left[1-\left(1/\lambda \right),\left(m+k\right){\left(\alpha /t\right)}^{\lambda }\right]}{\left[1-e^{-{\left(\alpha /x\right)}^{\lambda }}\right]e^{-\beta e^{-{\left(\alpha /x\right)}^{\lambda }}}}. \end{array}$$

### 3.7. Inequality Curves

For the NEXF distribution, the following Lorenz curves are defined:

(25) $$\begin{array}{c} L\left(p\right)=\frac{\Psi_{1}\left(x_{p}\right)}{\mu }=\frac{\sum_{m=0}^{1}\sum_{k=0}^{\infty }\Phi_{m,k}{\left(m+k\right)}^{s/\lambda }\gamma \left[1-\left(x_{p}/\lambda \right),\left(m+k\right){\left(\alpha /t\right)}^{\lambda }\right]}{\sum_{m=0}^{1}\sum_{k=0}^{\infty }\Phi_{m,k}\Gamma \left(1-\left(1/\lambda \right)\right)\left[\alpha {\left[m+k\right]}^{1/\lambda }\right]}, \end{array}$$

where *F*(*x*_*p*_)=*p*, Ψ_1_(*t*) is the first incomplete moment, and *x*_*p*_ is the quantile function.

Additionally, we can determine the Bonferroni and Zenga inequality curves based on the correlations to the Lorenz curve as shown in the following equation (for further details and further readings, see [34]):

(26) $$\begin{array}{c} B\left(p\right)=\frac{L\left(p\right)}{p},\\ Z\left(p\right)=\frac{L\left(p\right)-p}{p\left[1-L\left(p\right)\right]}. \end{array}$$

### 3.8. Order Statistics

For the *i* th order statistic of the NEXF distribution, the PDF and CDF are given as follows:

(27) fi:nx=n!i−1!n−i!Fxi−11−Fxn−ifx=λn!αλ1/xλ+1e−βe−α/xλ−2α/xλβ+1eα/xλ−βe−α/xλ−1eβ−e−α/xλ+1i−1ΓiΓ−i+n+1×e−α/xλ−1−eβ−e−α/xλn−i,Fi:nx=∑r=innrFxr1−Fxn−r=nie−α/xλ−1eβ−e−α/xλ+1ie−α/xλ−1−eβ−e−α/xλn−i×F121,i−n;i+1;1−eα/xλ+e−α/xλβ−1+eα/xλ,

where _2_*F*_1_(1, *i* − *n*; *i*+1; 1 − (*e*^(*α*/*x*)^*λ*^+*e*^−(*α*/*x*)^*λ*^^*β*^/−1+*e*^(*α*/*x*)^*λ*^^)) is a hypergeometric function.

## 4. Point Estimation Methods

This section is devoted to explain the different estimation methods that have been applied to to find the values of the estimates of the NEXF parameters according to two cases: firstly, a complete sample; secondly, Type-I censored samples. The estimation methods used are the maximum likelihood method (MLE) which is the most famous estimation technique to evaluate the parameters. Additionally, we used an important method of classical estimation which is the maximum product of spacing (MPS) method, and also we used the Bayesian estimation method depending on the squared error loss function.

### 4.1. Maximum Likelihood Method

Suppose that we have an order sample as following such that *x*_1_,…, *x*_*n*_ be a random sample from the NEXF distribution. This sample is based on the Type-I censored sample with vector parameter Θ=(*α*, *β*, *λ*), and the likelihood function of the NEXF distribution under the Type-I censored sample takes the form as follows:

(28) $$\begin{array}{c} L\left(\Theta \right)=c\lambda^{r}\alpha^{r}e^{-\sum_{i=1}^{r}{\left(\alpha /x_{i:n}\right)}^{\lambda }}e^{-\beta \sum_{i=1}^{r}e^{-{\left(\alpha /x_{i:n}\right)}^{\lambda }}}\prod_{i=1}^{r}{\left(\frac{\alpha }{x_{i:n}}\right)}^{\lambda -1}\left[1+\beta \left(1-e^{-{\left(\alpha /x_{i:n}\right)}^{\lambda }}\right)\right]{\left(\frac{1-e^{-{\left(\alpha /T\right)}^{\lambda }}}{e^{\beta e^{-{\left(\alpha /T\right)}^{\lambda }}}}\right)}^{n-r}, \end{array}$$

where *c* does not depend on parameters. The log-likelihood function of NEXF based on the Type-I censored sample takes the form as follows:

(29) $$\begin{array}{c} \ell \left(\Theta \right)\propto r\lambda \;\ln\left(\alpha \right)+r\;\ln\left(\lambda \right)-\left(\lambda -1\right)\overset{r}{\underset{i=1}{\sum }}\ln\left(x_{i:n}\right)-\overset{r}{\underset{i=1}{\sum }}{\left(\frac{\alpha }{x_{i:n}}\right)}^{\lambda }+\overset{r}{\underset{i=1}{\sum }}\ln\left[1+\beta \left(1-e^{-{\left(\alpha /x_{i:n}\right)}^{\lambda }}\right)\right]\\ -\beta \overset{r}{\underset{i=1}{\sum }}e^{-{\left(\alpha /x_{i:n}\right)}^{\lambda }}+\left(n-r\right)\ln\left(1-e^{-{\left(\alpha /T\right)}^{\lambda }}\right)-\left(n-r\right)\beta e^{-{\left(\alpha /T\right)}^{\lambda }}. \end{array}$$

Now, by differentiating the log-likelihood equation (29) with respect to *α*, *β*, and *λ* separately, we get the following equations:

(30) $$\begin{array}{c} \frac{\partial \ell \left(\Theta \right)}{\partial \alpha }=\frac{r\lambda }{\alpha }+\lambda \alpha^{\lambda -1}\overset{r}{\underset{i=1}{\sum }}{\left(\frac{1}{x_{i:n}}\right)}^{\lambda }+\beta \lambda \alpha^{\lambda -1}\overset{r}{\underset{i=1}{\sum }}\frac{e^{-{\left(1/x_{i:n}\right)}^{\lambda }}}{1+\beta \left(1-e^{-{\left(\alpha /x_{i:n}\right)}^{\lambda }}\right)} \end{array}$$

(31) $$\begin{array}{c} \frac{\partial \ell \left(\Theta \right)}{\partial \beta }=\overset{r}{\underset{i=1}{\sum }}\frac{\left(1-e^{-{\left(\alpha /x_{i:n}\right)}^{\lambda }}\right)}{1+\beta \left(1-e^{-{\left(\alpha /x_{i:n}\right)}^{\lambda }}\right)}-\overset{r}{\underset{i=1}{\sum }}e^{-{\left(\alpha /x_{i:n}\right)}^{\lambda }}-\left(n-r\right)e^{-{\left(\alpha /T\right)}^{\lambda }}=0, \end{array}$$

(32) $$\begin{array}{c} \frac{\partial \ell \left(\Theta \right)}{\partial \lambda }=\frac{r}{\lambda }-\overset{r}{\underset{i=1}{\sum }}\ln\left(x_{i:n}\right)+\overset{r}{\underset{i=1}{\sum }}{\left(\frac{\alpha }{x_{i:n}}\right)}^{\lambda }\ln\left(\frac{\alpha }{x_{i:n}}\right)\left(\beta e^{-{\left(\alpha /x_{i:n}\right)}^{\lambda }}-1\right)\\ +\beta \overset{r}{\underset{i=1}{\sum }}\frac{{\left(\alpha /x_{i:n}\right)}^{\lambda }\ln\left(\alpha /x_{i:n}\right)e^{-{\left(\alpha /x_{i:n}\right)}^{\lambda }}}{1+\beta \left(1-e^{-{\left(\alpha /x_{i:n}\right)}^{\lambda }}\right)}+\left(n-r\right)\frac{\ln\left(\alpha /T\right){\left(\alpha /T\right)}^{\lambda }e^{-{\left(\alpha /T\right)}^{\lambda }}}{1-e^{-{\left(\alpha /T\right)}^{\lambda }}}-\left(n-r\right)\beta \;\ln\left(\frac{\alpha }{T}\right){\left(\frac{\alpha }{T}\right)}^{\lambda }e^{-{\left(\alpha /T\right)}^{\lambda }}=0. \end{array}$$

Since the equations in (30)–(32) are not solved analytically, numerical approaches will be used to solve these equations such as the Newton–Raphson method.

### 4.2. The Maximum Product Spacing Method

In this subsection, we devoted our efforts to study the most famous classical method of estimation, namely, the MPS method which is considered as the first competitive for the MLEs. By referring to Ng et al. [35], Almetwally et al. [36], and Alshenawy et al. [37], the log-MPSEs under type-I censored samples for the NEXF distribution take the form as follows:

(33) $$\begin{array}{c} lS\left(\Theta \right)\propto \;\ln\left(1-\frac{1-e^{-{\left(\alpha /x_{1:n}\right)}^{\lambda }}}{e^{\beta e^{-{\left(\alpha /x_{1:n}\right)}^{\lambda }}}}\right)+\ln\left(\frac{1-e^{-{\left(\alpha /x_{r:n}\right)}^{\lambda }}}{e^{\beta e^{-{\left(\alpha /x_{r:n}\right)}^{\lambda }}}}\right)\\ +\overset{r}{\underset{i=2}{\sum }}\ln\left[\frac{1-e^{-{\left(\alpha /x_{i-1:n}\right)}^{\lambda }}}{e^{\beta e^{-{\left(\alpha /x_{i:n}\right)}^{\lambda }}}}-\frac{1-e^{-{\left(\alpha /x_{i:n}\right)}^{\lambda }}}{e^{\beta e^{-{\left(\alpha /x_{i:n}\right)}^{\lambda }}}}\right]+\left(n-r\right)\ln\left(\frac{1-e^{-{\left(\alpha /T\right)}^{\lambda }}}{e^{\beta e^{-{\left(\alpha /T\right)}^{\lambda }}}}\right). \end{array}$$

The MPSEs of distribution parameters for the Type-I censored samples can be derived through the following steps:

1. First derive the log-product equation (33)
2. Find the partial derivative for equation (33), with respect to each existing parameter, respectively
3. We all know that these equations are extremely tough to solve, so we will start here by using nonlinear optimisation algorithms such as the Newton–Raphson algorithm takes a role in solving these kinds of problems

### 4.3. Bayesian Estimation

This subsection presents Bayesian parameter estimations for the parameters based on the squared error (SE) loss function of the NEXF distribution parameters *α*, *β*, and *λ* based on the Type-I censored sample. The prior distributions of the parameters are chosen to be gamma distributions. Thus,

(34) $$\begin{array}{c} \pi_{1}\left(\alpha \right)\propto \alpha^{b_{1}-1}e^{-\alpha d_{1}},\;\alpha >0,b_{1},d_{1}>0,\\ \pi_{2}\left(\beta \right)\propto \beta^{b_{2}-1}e^{-\beta d_{2}},\;\beta >0,b_{2},d_{2}>0,\\ \pi_{3}\left(\lambda \right)\propto \lambda_{3}^{b_{3}-1}e^{-\lambda d_{3}},\;\lambda >0,b_{3},d_{3}>0. \end{array}$$

By presuming the independency of the proposed model parameters, we can get and formulate the joint PDF of the priors as follows:

(35) $$\begin{array}{c} \pi \left(\alpha ,\beta ,\lambda \right)\propto \alpha^{b_{1}-1}\beta^{b_{2}-1}\lambda^{b_{3}-1}e^{-\left(\alpha d_{1}+\beta d_{2}+\lambda d_{3}\right)}. \end{array}$$

Now, the posterior function of the proposed distribution's parameters may be calculated using equation (28) and also equation (35) as follows:

(36) $$\begin{array}{c} \pi^{*}\left(\Theta |x\right)\propto L\left(\alpha ,\beta ,\lambda \right)\pi \left(\alpha ,\beta ,\lambda \right)\\ \propto \alpha^{r+b_{1}-1}\beta^{b_{2}-1}\lambda^{r+b_{3}-1}e^{-\left(\alpha d_{1}+\lambda d_{3}\right)}e^{-\sum_{i=1}^{r}{\left(\alpha /x_{i:n}\right)}^{\lambda }}e^{-\beta \left(\sum_{i=1}^{r}e^{-{\left(\alpha /x_{i:n}\right)}^{\lambda }}+d_{2}\right)}\\ \prod_{i=1}^{r}{\left(\frac{\alpha }{x_{i:n}}\right)}^{\lambda -1}\left[1+\beta \left(1-e^{-{\left(\alpha /x_{i:n}\right)}^{\lambda }}\right)\right]{\left(\frac{1-e^{-{\left(\alpha /T\right)}^{\lambda }}}{e^{\beta e^{-{\left(\alpha /T\right)}^{\lambda }}}}\right)}^{n-r}. \end{array}$$

Bayesian parameter estimation for the NEXF distribution using the SE loss function is given by

(37) $$\begin{array}{c} {\tilde{\alpha }}_{\text{SE}}=\int_{0}^{\infty }\alpha \int_{0}^{\infty }\int_{0}^{\infty }\pi^{*}\left(\Theta |x\right)\text{d}\beta \text{d}\lambda \text{d}\alpha , \end{array}$$

(38) $$\begin{array}{c} {\tilde{\beta }}_{\text{SE}}=\int_{0}^{\infty }\beta \int_{0}^{\infty }\int_{0}^{\infty }\pi^{*}\left(\Theta |x\right)\text{d}\lambda \text{d}\alpha \text{d}\beta , \end{array}$$

(39) $$\begin{array}{c} {\tilde{\lambda }}_{\text{SE}}=\int_{0}^{\infty }\lambda \int_{0}^{\infty }\int_{0}^{\infty }\pi^{*}\left(\Theta |x\right)\text{d}\alpha \text{d}\beta \text{d}\lambda . \end{array}$$

It is very clear that the integrals in equations (37), (38) and (39) are complicated. Consequently, the Markov Chain Monte Carlo (MCMC) and Metropolis-Hastings (MH) algorithm are applied to obtain approximations for these integrals.

#### 4.3.1. Markov Chain Monte Carlo Technique

Multiple integrals, as we all know, are incredibly difficult to solve analytically or even mathematically by hand. To find an estimate for these integrals, we must use the MCMC technique. The MH algorithm, also known as the random walk algorithm, is an integral part of the MCMC technique. It is very similar to the process of acceptance and rejection sampling (Algorithm 1).

We can find the BEs of the distribution parameters *u*(*α*, *β*, *λ*) by the aid of the MH algorithm under the SE loss function, as follows:

(40) $$\begin{array}{c} {\tilde{u}}_{\text{SE}}=\frac{1}{N-M}\overset{N}{\underset{i=M+1}{\sum }}u\left(\alpha^{\left(i\right)},\beta^{\left(i\right)},\lambda^{\left(i\right)}\right). \end{array}$$

## 5. Interval Estimation for the Distribution's Parameters

This part of the paper was devoted for interval estimation as we performed interval estimation for the distribution parameters according to two methods: the asymptotic and Credible CIs methods.

### 5.1. Asymptotic Confidence Intervals

Asymptotic CI is the most popular approach to establishing approximate confidence limits for parameters, in which MLEs are used to get the Fisher information matrix $I\left(\hat{\Omega }\right)$, which consists of the second derivative with negative signs for the log-likelihood function, where we substitute with the estimates of the MLEs $\hat{\Omega }=\left(\hat{\alpha },\hat{\beta },\hat{\lambda }\right)$, where

(41) $$\begin{array}{c} I\left(\hat{\Omega }\right)=\left[\begin{array}{ccc} I_{\hat{\alpha }\hat{\alpha }} & \; & \;\\ I_{\hat{\beta }\hat{\alpha }} & I_{\hat{\beta }\hat{\beta }} & \;\\ I_{\hat{\beta }\hat{\lambda }} & I_{\hat{\alpha }\hat{\lambda }} & I_{\hat{\lambda }\hat{\lambda }} \end{array}\right]. \end{array}$$

In order to find the asymptotic variance-covariance matrix, we get the inverse matrix for the Fisher information matrix. We have the vector parameter Ω as $V\left(\hat{\Omega }\right)=I^{-1}\left(\hat{\Omega }\right)$.

So, the 100(1 − *γ*)% asymptotic CI for the parameters *α*, *β*, and *λ* can be established as follows:

(42) $$\begin{array}{c} \left({\hat{\vartheta }}_{l},{\hat{\vartheta }}_{u}\right)=\hat{\vartheta }\pm Z_{1-\gamma /2}\sqrt{V\left(\hat{\vartheta }\right)}, \end{array}$$

where *ϑ* is *α*,  *λ*, and *β* are the parameters of the distribution and *Z*_*q*_ is the 100*q* − th which is the the standard normal distribution's percentile.

### 5.2. Highest Posterior Density (HPD) Interval Algorithm

According to Bayesian estimation, we find point and interval estimations so we must find interval estimation for the distribution's parameter. This interval is called the HPD interval or sometimes the credible intervals. We explained the technique for discovering the (1 − *γ*) HPD interval for *α*, *β*,  and *λ*. This method has been suggested by [38] (Algorithm 2).

## 6. Simulation Study

As of now, for any distribution, we must evaluate its performance by using different values for its parameters so we must perform a simulation study under both a complete and a Type-I censored sample. The Monte Carlo simulation is conducted in this section to compare the performance of the methods used in the paper and determine the behaviours of the parameters using the MLEs, MPS, and Bayesian estimates of the NEXF parameters under Type-I censored samples, as depending on the R programming. Ten thousand random samples were generated from the NEXF distribution according to the following combinations of parameters.

We used different values for the parameters with different combination as shown in Tables 1–4 , with varying sample sizes as shown in the following tables and different time point *T* to end the experiment. In the results of the CI, *γ* is chosen to be 0.05. We may define the optimal approach as one that minimises bias, mean squared error (MSE), and length of the confidence interval (L.CI) of the estimator. Comparing the results of the point estimation depends on the bias, MSE, and L.CI values. Tables 1–4 show the different results of simulating the point estimation methods suggested throughout this paper.

### 6.1. Concluding Remarks Conducted from the Simulation Study

The following observations can be easily conducted from the results conducted from the simulation. We used Algorithms 1 and 2 to get the simulation results.

1. As the sample size increases, the MSE, Bias, and CI length of each of the parameters decrease, which is the consistence property
2. As the censoring time of Type-I (*T*) increases, the value of the Bias is decreased
3. As the censoring time of Type-I (*T*) increases, the value of the MSE is also decreased
4. As the censoring time of Type-I (*T*) increases, the value of the Length of CI is also decreased
5. In most cases, the MPS performs in a better case than MLE under Type-I censored samples
6. We concluded that the credible interval provides the smallest length among all CIs, when the sample is generated under Type-I censored sample
7. We can analyze that by increasing *λ*, the MSE and Bias and CI length for the parameter *α* decrease while for *β* increases, in most cases
8. We can analyze that by increasing *β*, the MSE and Bias and CI length for the parameter *α* decrease while for *λ* decreases, in most cases
9. We can analyze that by increasing *α*, the MSE and Bias and CI length for the parameter *λ* decrease while for *β* decreases, in most cases

## 7. Data Analysis Using Type-I Censored Data

In this part of the paper, we perform a real-world data analysis for type progressive censoring data. We used the new novel modified KS algorithm to fit the Type-I censored data.  Algorithm 3 discusses the steps for fitting Type-I censored data (see [39]).

### 7.1. Model Selection Criteria

The selection of models for specific data is one of the basic tasks of the scientific study in choosing a predictive model from a group of candidate models. Several statistical methods are available to determine the fitness of competing distributions, where the most widely used are the Akaike information criteria (AIC) and the Bayesian knowledge criteria (BIC). The optimal distribution for the real data set may be the one with the lowest values. These methods are determined according to the following formulas:

The AIC is given by

(43) $$\begin{array}{c} \text{AIC}=2k-2\ell . \end{array}$$

The CAIC is

(44) $$\begin{array}{c} \text{CAIC}=\frac{2nk}{n-k-1}-2\ell . \end{array}$$

The BIC is evaluated as follows:

(45) $$\begin{array}{c} \text{BIC}=k\;\log\left(n\right)-2\ell . \end{array}$$

The HQIC is

(46) $$\begin{array}{c} \text{HQIC}=2k\;\log\left(\log\left(n\right)\right)-2\ell , \end{array}$$

such that *ℓ* is the MLE log-likelihood function value, and *k* is parameters count in the distribution in the proposed model, and *n* is considered as the size of the sample used in calculations. We take the AIC and BIC tests to demonstrate that the distribution presented is the most appropriate fit for the data. In order to compare between a large number of distributions, we must base such a comparison on certain criteria: one of these information criteria is called the Akaike information criterion (AIC) (see Akaike [40]) though there are other criteria which are called the Bayesian information criterion (BIC) (see Schwarz [41] for more information), and we can also refer to the Hannan–Quinn criterion (for more information on the criterion (HQIC), see Hannan and Quinn [42]), and for more information and last criteria called the consistent Akaike information criterion (CAIC), refer to the study by Bozdogan [43]; all these criteria were used to determine which model among all competing ones is the best for statistical modeling of the data.

### 7.2. Real Data Set Application for Remission Times

This subsection includes a data analysis to demonstrate the distribution's performance. We can find these data in Bain and Engelhardt [44]. This data represent how long leukaemia patients survive with a new treatment for each patient. We recorded the remission times of leukaemia patients after using a new drug for treatment. The new medication that leads to remission in leukaemia was given to a group of 40 patients; after seven months (210 days), the trial was then terminated. It is obvious that we have a Type-I censored sample with *n*=40 and *m*=22, where *m* donates the number of recorder times before the experiments reach an end and *T*=205, where *T* is the time at which the experiments ended.

To verify that the likelihood function exists and has unique values for its estimates, the existence and uniqueness property is studied as it is very important property that proves that the likelihood function has unique and global maximum roots, and the likelihood function is plotted in Figures 3 and 4 , respectively.  Figure 3 confirms the existence of MLEs as the derivative of the log-likelihood function with respect to a certain parameter that intersects the *x*-axis at a single point. In addition, Figure 4 provides the truth that estimates for the parameters are global maximum roots. Obviously, the log-likelihood function is a decreasing function that crosses the *x*-axis only once. As a result, we can assert that the log-likelihood function has only one unique root, which is the global maximum.

The results in the tables show the values of the parameters and the goodness of fit criteria values for the proposed distribution in the competition that were used in the comparison; in this section, we introduce the competitive distributions used in comparison with our proposed model.  Table 5 is concerned with the parameter estimation of the distribution's parameters.  Table 6 is concerned with the values of AIC, BIC, HQIC, and and CAIC of the distributions. We compare the proposed distribution with the Exponential distribution (E), CDF=*e*^−(*x*/*λ*)^−*α*^^, Fréchet two-parameter distribution (F), CDF=1 − (1 − exp(−(*α*/*x*)^*λ*^)/exp(*β*  exp(−(*α*/*x*)^*λ*^))), and the Fréchet three parameters distribution (FTP), CDF=*e*^−(*x* − *μ*/*β*)^−*α*^^.

## 8. Conclusions and Remarks

A new novel model has been studied and introduced in this paper, and this model called the NEXF distribution. Its statistical properties have been studied and a linear representation is obtained which helps to find the moments and generating functions. The three unknown parameters of the NEXF distribution have been estimated using the classical and Bayesian approaches of estimation under complete and Type-I censoring schemes. Simulations were performed to test the efficiency of the estimation methods. The MH algorithm has a great role for obtaining an approximation for the Bayesian estimates. We can easily conduct from the results tabulated in the simulation section that the Bayesian method performs better than the other methods according to the values of the MSE. From the real data example, we can see that the NEXF distribution is the best fit of data than the E, F, and FTP distributions. We used the modified KS test to determine the goodness of fit for each distribution to the data. Also, we discussed the existence and uniqueness of the log-likelihood function graphically. We proved that the roots maximize the log-likelihood function and also proved that these roots are unique, and at last we proved the superiority of the proposed distribution in modeling and fitting healthcare and medical data.

## Figures and Tables

**Figure 1:** PDF plots of NEXF distribution.

**Figure 2:** HRF plots of NEXF distribution.

**Figure 3:** The uniqueness of the roots of the log-likelihood.

**Figure 4:** The log-likelihood roots being global maximum.

**Algorithm 1:** The MH algorithm can be known as an approximation method for evaluating integrals that cannot be evaluated explicitly.

**Algorithm 2:** Credible interval algorithm.

**Algorithm 3:** Fitting Type-I censored data using a modified KS algorithm.

**Table 1:** MLE, MPS, and Bayesian estimations of the NEXF distribution parameters under the complete sample when *α*=0.5.

*α*=0.5				MLE			MPS			Bayesian		
*β*	*λ*	*n*		Bias	MSE	L.CI	Bias	MSE	L.CI	Bias	MSE	L.CCI
0.5	0.5	50	*α*	0.0991	0.1998	1.7102	0.0967	0.0721	0.9826	0.0914	0.0662	0.8906
			*β*	0.0226	0.5260	2.8444	0.1115	0.1582	1.4981	0.0473	0.1335	1.2607
			*λ*	0.0442	0.0108	0.3687	−0.0142	0.0050	0.2705	0.0055	0.0043	0.2571
		100	*α*	−0.0055	0.1149	1.3300	0.0189	0.0245	0.6099	0.0688	0.0413	0.6820
			*β*	−0.1086	0.3453	2.2661	0.0048	0.0522	0.8961	0.0377	0.1191	1.1571
			*λ*	0.0177	0.0070	0.3219	−0.0229	0.0031	0.1994	0.0004	0.0022	0.1875
		200	*α*	−0.0185	0.0423	0.8041	0.0350	0.0196	0.5316	0.0551	0.0369	0.6119
			*β*	−0.1067	0.1989	1.6989	0.0407	0.0553	0.9092	0.0245	0.0920	1.0364
			*λ*	0.0248	0.0045	0.2446	−0.0088	0.0017	0.1595	0.0027	0.0016	0.1572
	3	50	*α*	−0.0036	0.0021	0.1802	0.0031	0.0009	0.1195	0.1072	0.0021	0.1451
			*β*	−0.1102	1.4597	4.7187	0.0288	0.0870	1.1515	0.2854	0.9675	2.5970
			*λ*	0.1221	0.3848	2.3852	−0.1361	0.0942	1.0785	−0.3356	0.3570	2.0606
		100	*α*	−0.0026	0.0019	0.1724	0.0016	0.0004	0.0800	0.0722	0.0017	0.1683
			*β*	−0.0498	0.9000	3.7156	0.0227	0.0492	0.8656	0.1960	0.4585	1.8786
			*λ*	0.0559	0.1295	1.3945	−0.0960	0.0479	0.7716	−0.0833	0.1247	1.3434
		200	*α*	0.0010	0.0004	0.0747	0.0019	0.0002	0.0556	0.0167	0.0004	0.0685
			*β*	0.0064	0.2402	0.9786	0.0159	0.0283	0.6568	0.1409	0.0305	0.6539
			*λ*	0.0147	0.0277	0.6501	−0.0565	0.0224	0.5438	0.0076	0.0116	0.6025

3	0.5	50	*α*	0.0382	0.0895	1.1661	0.0788	0.0583	0.8965	0.0361	0.0714	1.1289
			*β*	−0.0373	0.3105	2.9476	−0.0009	0.1392	1.4664	0.0147	0.9626	2.5120
			*λ*	0.0271	0.0067	0.3034	−0.0120	0.0028	0.2012	0.0314	0.0060	0.2931
		100	*α*	0.0327	0.0416	0.7909	0.0593	0.0287	0.6241	0.0295	0.0389	0.7091
			*β*	−0.1022	0.2209	2.5176	0.0148	0.1025	1.2571	0.0038	0.1903	2.0657
			*λ*	0.0124	0.0028	0.2005	−0.0107	0.0012	0.1278	0.0116	0.0024	0.1985
		200	*α*	0.0067	0.0354	0.7384	0.0471	0.0181	0.4957	0.0689	0.0342	0.6779
			*β*	0.0103	0.1538	1.5405	0.0502	0.0721	1.0364	0.0162	0.1469	1.3696
			*λ*	0.0057	0.0014	0.1450	−0.0087	0.0007	0.0999	0.0048	0.0010	0.1170
	3	50	*α*	−0.0040	0.0015	0.1517	0.0000	0.0003	0.0644	−0.0027	0.0015	0.1469
			*β*	−0.0405	0.4085	4.6612	−0.0147	0.0045	0.2571	0.0374	0.4069	4.1761
			*λ*	0.1818	0.5542	2.8369	−0.0434	0.0312	0.6726	0.2568	0.3927	2.0036
		100	*α*	0.0022	0.0003	0.0619	0.0015	0.0001	0.0442	0.0015	0.0002	0.0513
			*β*	0.0131	0.0274	0.6489	−0.0140	0.0016	0.1488	0.0297	0.0100	3.6953
			*λ*	−0.0007	0.0413	0.7989	−0.0455	0.0115	0.3812	0.0100	0.0416	0.7496
		200	*α*	−0.0015	0.0007	0.0320	0.0007	0.0001	0.0298	0.0006	0.0005	0.0881
			*β*	−0.0097	0.0061	0.1925	−0.0075	0.0007	0.0992	0.0036	0.0059	0.1676
			*λ*	0.0251	0.0145	0.3670	−0.0293	0.0056	0.2703	0.0142	0.0125	0.2863

**Table 2:** MLE, MPS, and Bayesian estimations of the NEXF distribution parameters under the complete sample when *α*=3.

*α*=3				MLE			MPS			Bayesian		
*β*	*λ*	*n*		Bias	MSE	L.CI	Bias	MSE	L.CI	Bias	MSE	L.CCI
0.5	0.5	50	*α*	−0.1484	0.7181	3.2721	0.1119	0.1103	1.2266	0.1361	0.6878	3.0497
			*β*	−0.0873	0.1978	1.7102	0.0457	0.0864	1.1388	0.0507	0.1419	1.2495
			*λ*	0.0296	0.0071	0.3099	−0.0217	0.0031	0.2008	−0.0007	0.0068	0.2811
		100	*α*	−0.1831	1.0738	4.0001	0.0895	0.0475	0.7798	0.1401	1.0118	3.9270
			*β*	−0.1116	0.2084	1.7363	0.0419	0.0447	0.8132	0.0284	0.1004	1.0719
			*λ*	0.0223	0.0041	0.2351	−0.0163	0.0015	0.1391	0.0018	0.0021	0.1765
		200	*α*	−0.2206	0.5232	2.7015	0.0521	0.0210	0.5307	0.1933	0.4953	2.6839
			*β*	−0.1149	0.1169	1.2633	0.0144	0.0218	0.5764	0.0227	0.0856	1.0496
			*λ*	0.0169	0.0026	0.1872	−0.0103	0.0007	0.0985	0.0000	0.0013	0.1413
	3	50	*α*	0.0040	0.2771	2.0646	0.1089	0.1555	1.4862	0.0041	0.0268	0.6570
			*β*	−0.0424	1.5094	3.8931	0.2460	0.6146	2.9194	0.0106	0.1025	1.0786
			*λ*	0.1368	0.4123	2.4606	−0.2261	0.2708	1.8382	0.0324	0.0894	1.1261
		100	*α*	0.0207	0.2564	1.9845	0.1156	0.1027	1.1726	0.0010	0.0205	0.5611
			*β*	−0.1123	0.9161	3.2645	0.2385	0.4124	2.3384	−0.0089	0.0813	1.0053
			*λ*	0.0865	0.3400	2.2615	−0.1828	0.1735	1.4678	0.0346	0.0510	0.9074
		200	*α*	−0.0411	0.1779	1.6511	0.0700	0.0532	0.8643	0.0055	0.0175	0.4788
			*β*	−0.1049	0.8313	2.8274	0.1424	0.2198	1.7567	0.0079	0.0782	0.9221
			*λ*	0.0544	0.2230	1.8451	−0.1381	0.1144	1.2140	−0.0039	0.0353	0.6828

3	0.5	50	*α*	0.0147	1.5829	4.9339	0.0218	0.0916	1.1837	0.0434	0.9236	4.0988
			*β*	0.0019	1.2477	4.3809	−0.1030	0.1326	1.3697	0.0021	0.9746	4.0213
			*λ*	0.0276	0.0073	0.3176	−0.0135	0.0022	0.1740	0.0142	0.0070	0.3084
		100	*α*	−0.1704	0.6306	3.0420	0.0177	0.0344	0.7241	0.1383	0.6084	2.8996
			*β*	−0.1406	0.5735	2.9184	−0.0397	0.0513	0.8742	0.0919	0.4851	2.7985
			*λ*	0.0268	0.0053	0.2656	−0.0084	0.0009	0.1156	0.0188	0.0050	0.2718
		200	*α*	0.1542	0.4663	2.6091	0.0111	0.0168	0.5063	0.1250	0.2167	2.2144
			*β*	0.1239	0.2653	1.9607	−0.0234	0.0266	0.6333	0.0286	0.2166	1.6485
			*λ*	−0.0005	0.0011	0.1287	−0.0059	0.0005	0.0829	0.0016	0.0010	0.1245
	3	50	*α*	−0.0487	0.5327	2.8650	0.0127	0.0338	0.7212	0.0043	0.0745	0.8985
			*β*	−0.3755	1.3831	4.5835	−0.0129	0.3712	2.3967	0.1552	0.9005	3.9774
			*λ*	0.2343	0.3604	4.0067	−0.0564	0.1218	1.3550	0.1824	0.2720	2.0924
		100	*α*	0.0393	0.1632	1.5768	0.0217	0.0181	0.5210	0.0224	0.1549	0.8250
			*β*	0.0262	0.7696	3.3472	0.0208	0.2204	1.8395	0.0225	0.2213	1.8356
			*λ*	0.0957	0.1750	2.3723	−0.0716	0.0725	1.0179	0.0939	0.1644	1.5120
		200	*α*	0.0186	0.1486	1.4688	0.0228	0.0177	0.5135	0.0142	0.0861	0.8066
			*β*	−0.0606	0.2954	1.9300	0.0174	0.2112	1.8011	0.0595	0.1898	4.1254
			*λ*	0.1084	0.3983	2.4384	−0.0748	0.0696	0.9923	0.0865	0.1560	1.5026

**Table 3:** MLE, MPS, and Bayesian estimations of the NEXF distribution parameters under the Type-I censored sample when *α*=0.5 and *β*=0.5.

				MLE			MPS			Bayesian		
*λ*	*T*	*n*		Bias	MSE	L.CI	Bias	MSE	L.CI	Bias	MSE	L.CCI
0.5	1.5	50	*α*	0.0331	0.1879	1.6951	0.1233	0.0857	1.0413	0.0811	0.0494	0.7536
			*β*	−0.1455	0.5428	2.8325	0.1338	0.2140	1.7367	0.0432	0.1130	1.1443
			*λ*	0.0420	0.0114	0.3859	−0.0276	0.0058	0.2791	0.0052	0.0031	0.2030
		100	*α*	0.0559	0.1506	1.5060	0.1154	0.0593	0.8410	0.0551	0.0334	0.6300
			*β*	−0.0864	0.5040	2.7637	0.1350	0.1428	1.3842	0.0084	0.0752	0.9128
			*λ*	0.0187	0.0067	0.3136	−0.0283	0.0034	0.2008	0.0011	0.0021	0.1478
		200	*α*	−0.0275	0.0401	0.7777	0.0876	0.0338	0.6338	0.0558	0.0387	0.6305
			*β*	−0.1353	0.2322	1.8141	0.1360	0.0924	1.0659	0.0380	0.0858	1.0452
			*λ*	0.0202	0.0038	0.2294	−0.0215	0.0019	0.1474	−0.0014	0.0012	0.1374
	2.5	50	*α*	0.0615	0.1755	1.6262	0.0502	0.0316	0.6693	0.1074	0.0779	0.9053
			*β*	−0.0443	0.3909	2.4472	0.0288	0.0429	0.8045	0.0295	0.1092	1.0853
			*λ*	0.0313	0.0096	0.3641	−0.0206	0.0043	0.2443	0.0042	0.0036	0.2263
		100	*α*	0.0924	0.1985	1.7104	0.0590	0.0577	0.9137	0.0750	0.0453	0.7297
			*β*	0.0113	0.5141	2.8130	0.0578	0.1404	1.4527	0.0502	0.1041	1.0816
			*λ*	0.0195	0.0080	0.3423	−0.0145	0.0037	0.2314	−0.0009	0.0020	0.1705
		200	*α*	−0.0124	0.0435	0.8166	0.0303	0.0130	0.4318	0.0562	0.0372	0.6233
			*β*	−0.0978	0.2144	1.7761	0.0367	0.0431	0.8016	0.0324	0.0942	1.0172
			*λ*	0.0209	0.0040	0.2332	−0.0103	0.0013	0.1372	0.0007	0.0014	0.1456

3	0.5	50	*α*	−0.0027	0.0023	0.1875	−0.0018	0.0005	0.0866	0.0134	0.0022	0.1780
			*β*	−0.0646	0.9606	3.8375	−0.0508	0.0375	0.7334	0.0167	0.1399	1.2548
			*λ*	0.1420	0.3803	2.3547	−0.1000	0.0805	1.0418	−0.0045	0.2804	2.0021
		100	*α*	−0.0054	0.0032	0.2214	0.0015	0.0007	0.1005	0.0048	0.0012	0.1260
			*β*	−0.1203	1.5305	4.8315	−0.0167	0.0664	1.0089	0.0003	0.1199	1.1584
			*λ*	0.0772	0.2004	1.7301	−0.1052	0.0685	0.9404	0.0082	0.1411	1.4911
		200	*α*	0.0006	0.0003	0.0666	−0.0014	0.0001	0.0415	−0.0004	0.0003	0.0649
			*β*	0.0184	0.0316	0.6943	−0.0283	0.0071	0.3126	−0.0139	0.0251	0.6514
			*λ*	0.0095	0.0313	0.6937	−0.0537	0.0173	0.4717	0.0084	0.0280	0.6708
	1	50	*α*	−0.0007	0.0013	0.1426	−0.0022	0.0004	0.0804	0.0062	0.0012	0.1325
			*β*	−0.0371	0.6561	3.1750	−0.0304	0.0228	0.5805	0.0146	0.1244	1.1268
			*λ*	0.0951	0.1672	1.5605	−0.0732	0.0506	0.8348	0.0282	0.1281	1.3599
		100	*α*	−0.0002	0.0014	0.1488	0.0021	0.0007	0.1040	0.0016	0.0008	0.1097
			*β*	−0.0261	0.9689	3.8611	0.0323	0.0596	0.9496	0.0026	0.1134	1.1460
			*λ*	0.0707	0.1745	1.6155	−0.0635	0.0541	0.8784	0.0363	0.0813	1.0865
		200	*α*	0.0012	0.0004	0.0812	−0.0009	0.0002	0.0508	−0.0005	0.0004	0.0594
			*β*	0.0172	0.0316	0.6738	−0.0086	0.0063	0.3096	−0.0101	0.0286	0.6018
			*λ*	0.0116	0.0272	0.6450	−0.0366	0.0143	0.4465	0.0063	0.0255	0.6591

**Table 4:** MLE, MPS, and Bayesian estimations of the NEXF distribution parameters under Type-I censored sample when *α*=0.5 and *β*=3.

				MLE			MPS			Bayesian		
*λ*	*T*	*n*		Bias	MSE	L.CI	Bias	MSE	L.CI	Bias	MSE	L.CCI
0.5	0.5	50	*α*	−0.0373	0.0931	1.1880	0.0361	0.0446	0.8166	0.0894	0.0763	0.8930
			*β*	−0.3584	2.4411	5.9673	−0.1088	0.5360	2.8409	0.2132	1.7603	4.9731
			*λ*	0.0662	0.0178	0.4543	−0.0036	0.0060	0.3035	0.0230	0.0059	0.2633
		100	*α*	−0.0520	0.0270	0.6120	0.0143	0.0125	0.4356	0.0573	0.0691	0.9451
			*β*	−0.2964	0.7370	3.1616	−0.0302	0.0747	1.0661	0.0501	1.3972	4.5919
			*λ*	0.0390	0.0072	0.2967	−0.0050	0.0023	0.1859	0.0289	0.0059	0.2676
		200	*α*	0.0439	0.0344	0.7074	0.0569	0.0263	0.5965	0.0665	0.0539	0.8346
			*β*	0.1434	0.6359	3.0780	0.1502	0.2877	2.0204	0.0952	1.0236	3.8831
			*λ*	0.0029	0.0024	0.1922	−0.0116	0.0016	0.1481	0.0157	0.0039	0.2316
	1	50	*α*	−0.0209	0.0882	1.1621	0.0344	0.0415	0.8069	0.0860	0.0739	0.8201
			*β*	−0.2746	1.8209	5.1842	−0.0587	0.5109	2.7951	0.2130	1.4807	4.6516
			*λ*	0.0615	0.0187	0.4788	−0.0047	0.0060	0.3016	0.0209	0.0057	0.2730
		100	*α*	−0.0233	0.0266	0.6337	0.0308	0.0124	0.4246	0.0654	0.0249	0.7580
			*β*	−0.2472	0.6578	3.0310	−0.0227	0.0594	0.9524	0.0404	0.6588	3.0679
			*λ*	0.0281	0.0063	0.2920	−0.0125	0.0023	0.1822	0.0165	0.0037	0.2206
		200	*α*	0.0404	0.0339	0.6959	0.0526	0.0257	0.5860	0.0363	0.0304	0.6702
			*β*	0.1201	0.6270	3.0253	0.1458	0.2834	2.0211	0.1203	0.5713	3.0310
			*λ*	0.0026	0.0022	0.1902	−0.0110	0.0016	0.1358	0.0096	0.0021	0.1815

3	0.4	50	*α*	−0.0057	0.0037	0.2390	0.0153	0.0012	0.1238	0.0123	0.0056	0.2450
			*β*	−0.5002	1.9739	6.9792	−0.0474	0.0167	0.4716	0.1460	1.1515	4.2750
			*λ*	0.1775	0.9834	3.8284	−0.1972	0.1494	1.3047	0.1637	0.5406	2.7781
		100	*α*	0.0024	0.0004	0.0789	0.0056	0.0004	0.0755	0.0016	0.0033	0.1893
			*β*	−0.0091	0.0351	0.7342	−0.0177	0.0031	0.2061	0.0675	0.0349	0.7809
			*λ*	−0.0040	0.0697	1.0355	−0.0959	0.0477	0.7701	0.1398	0.2364	1.7967
		200	*α*	−0.0148	0.0059	0.2952	0.0040	0.0003	0.0636	−0.0007	0.0021	0.1744
			*β*	−0.2604	0.9021	4.5265	0.0350	0.1257	1.3843	0.1488	0.4470	2.5690
			*λ*	0.1566	0.4446	2.5432	−0.0556	0.0477	0.8289	0.1425	0.2274	1.8035
	0.8	50	*α*	−0.0012	0.0016	0.1576	0.0038	0.0005	0.0823	−0.0012	0.0018	0.1739
			*β*	0.0212	1.3022	4.4770	−0.0216	0.0398	0.7777	0.0741	1.8630	4.9506
			*λ*	0.1070	0.1981	1.6952	−0.0869	0.0756	1.0239	0.2244	0.3381	1.9961
		100	*α*	−0.0002	0.0005	0.0866	0.0005	0.0002	0.0485	0.0000	0.0009	0.1189
			*β*	0.0190	0.2223	1.8484	−0.0124	0.0063	0.3086	0.0837	0.8882	3.6324
			*λ*	0.0238	0.0658	1.0023	−0.0493	0.0198	0.5164	0.0984	0.1263	1.3225
		200	*α*	−0.0070	0.0043	0.2547	0.0033	0.0003	0.0691	0.0006	0.0004	0.0784
			*β*	−0.2034	0.8296	3.5845	0.0184	0.1815	1.6701	0.0339	0.3728	2.3717
			*λ*	0.1154	0.5351	2.8344	−0.0515	0.0418	0.7767	0.0475	0.0484	0.8331

**Table 5:** The MLEs for the distribution parameters used in the data analysis.

6 Distribution	$\hat{\alpha }$	*β*	*λ*
E	—	—	0.00329588
F	1.27842	—	151.189
FTP	0.733672	56.8345	42.2071
NEXF	14933.1	120.539	0.37816

**Table 6:** AIC, BIC, HQIC, and CAIC of the distributions.

Distribution	AIC	CAIC	BIC	HQIC	KS	*P* value
E	297.464	297.569	299.152	298.0744	0.169182	0.1095
F	288.518	288.842	291.895	289.739	0.115193	0.4475
FTP	300.488	301.155	305.554	302.32	0.301	0.001
NEXF	288.008	288.67	293.07	289.843	0.085467	0.7756

## Data Availability

All data are included within the paper, all references for all data are included in the paper, and all links and references are included in the paper.
